The article "Comparative Analysis of Female Leadership Styles in Public and Private Sector Universities: A Study in Pakistan" was retracted in 2025. Reason: plagiarism.

# Comparative Analysis of Female Leadership Styles in Public and Private Sector Universities: A Study in Pakistan

**DOI:** 10.1016/j.heliyon.2023.e22058

**Published:** 2023-11-10

**Authors:** Uzma Sarwar, Rameez Tariq, Muhammad Aamir, Yurong Guan

**Affiliations:** a School of Education, Huanggang Normal University, Huanggang, 438000 PR China; b Department of Management Sciences, COMSATS University, Islamabad, Park Road, Tarlai Kalan Islamabad 45550, Pakistan; c College of Computer Sciences, Huanggang Normal University, Huanggang, 438000 PR China

**Keywords:** Leadership style, Transformational, Transactional, Pakistan

## Abstract

This study aimed to compare the styles of leadership practices of female leaders in public and private Universities in Pakistan. In this study, both quantitative and qualitative data were collected using a mixed-method approach. An adapted and developed questionnaire was used for quantitative data collection, whereas qualitative data were collected through a semi-structured interview schedule. A sample of 200 female leaders was selected for quantitative data collection, while 10 females from the said sample were selected for qualitative data collection through a simple random method. Quantitative data were analyzed using SPSS, whereas qualitative data were analyzed using thematic analysis. Based on the statistical results, this study discovered statistically significant differences in female transformational and transactional leadership styles and significant differences in job performance based on the university sector. This study discovered statistically insignificant differences based on the different positions of female leaders regarding transformational and transactional leadership, and job performance. Moreover, qualitative data revealed that female leaders clearly understood both leadership styles and how to improve job performance by practicing them. The originality of this study concerns the identification of the differences between leadership styles (transformational and transactional) practiced by female leaders of public and private Universities in Pakistan and explains female leaders' perceptions of the role of leadership styles in their job performance.

## 1 Introduction

Recent studies have shown that both the transformational and transactional leadership styles are widely accepted. This has led many scholars to study organizational development and leaders' performance in leadership situations, with many challenges to become interested in these styles [[1], [2], [3]]. Research has shown that both transformational and transactional leadership have a positive effect on employee job performance [[3], [4], [5]]. [6] found that women in leadership positions have the potential to improve a company's success, particularly in terms of sales, quality of products and services in the light of a new meta-analysis that looked at the impact of women's participation in organizational leadership roles on financial performance.

The article "Comparative Analysis of Female Leadership Styles in Public and Private Sector Universities: A Study in Pakistan" was retracted in 2025. Reason: plagiarism.

Leadership is the ability to inspire others to take action in pursuit of a shared objective [7]. A leadership style is a method of leading an organization to succeed through the dissemination of vision, execution of strategies, and inspiration of its members [8]. According to Ref. [9]; leadership style is one of the most influential aspects of an organization's productivity and success. Northhouse (2016) argues that an organization's leadership may be defined as an individual's capacity to persuade other people to work together toward a shared objective. To lead effectively, one must be able to make tough decisions, communicate an inspiring vision, set realistic goals, and empower followers to achieve these goals [10]. Self-assurance, strong communication and management skills, originality of thought, resilience in the face of setbacks, willingness to take risks, and adaptability are all hallmarks of a successful leader [11]. Different types of political, business, and educational leaders use different tactics (Nanjundeswaraswamy & Swamy, 2014).

An organization needs strong leadership to achieve its vision, purpose, and objectives that can devise successful strategies, policies, and methods of action, as well as guide and coordinate the work of its members [12]. According to Harris et al. (2017), leadership of the highest quality is needed to achieve the mission and vision and deal with changes in the external environment. Many organizations face trouble because of unethical behavior, high employee turnover, bad financial performance, and so on. This could be because the people in charge were not doing a good job. The main goal of many organizations is to reach their goals, so they need good leaders to keep everyone on the same page and motivate them (Vigoda-Gadot, 2017). It is the most crucial element in an organization and the most crucial talent for the leaders of the company, as stated by Ref. [13]. The performance of an employee is affected both directly and indirectly. According to Ref. [14]; leadership is essential for fostering a culture that promotes information sharing, staff retention, and brand loyalty. Bass and Avolio proposed the Full Range Leadership paradigm in 1994 (FRL). The model showed that transformational and transactional leadership styles were the most effective. According to the FRL model, using both leadership philosophies at once impacts subordinates' attitudes and behavior, motivating them to improve their performance. The FRL model has been proven to work in various contexts including Korea, the United Kingdom, and Thailand [15,16]. Several ideas have been developed to explain successful leadership. Overall, workers’ effectiveness is closely correlated with transformational and transactional leadership styles (Kirkman, Chen, Farh, Chen, & Lowe, 2019).

The article "Comparative Analysis of Female Leadership Styles in Public and Private Sector Universities: A Study in Pakistan" was retracted in 2025. Reason: plagiarism.

However, despite 75 years of independence, Pakistan's educational system is still struggling with many issues, including inadequate leadership, and has not managed to reach its objectives and intended aims for quality education [17]. UNDP reports that Pakistan ranks 154th out of 189 nations in the Human Development Index (HDI) in 2020 [18]. According to the Pakistan Economic Survey (2019), the literacy rate in Pakistan is 57 %, and 43 % of the population is still illiterate [17]. states that the quality of education at private universities is better than that at public universities. It is believed that the way leaders of private universities run their schools is better than the way leaders of public universities run their schools. Moreover, according to Ref. [19]; the credibility of higher education institutions is based on several factors. However, leadership is generally thought to be the most important of all the leadership styles. Similarly, leadership styles have been considered a possible and essential predictor of different organizational outcomes. Transformational and transactional leadership styles are important for employee job performance. Similarly, employee performance is the only variable that determines the success or failure of organizations, including higher education institutions (HEIs).

Unfortunately, most schools and universities do not care about the management style of their top officials. Based on this assumption, the current study seeks to examine the leadership styles of women in the public and private university sectors and to learn how these women perceive their leadership styles to influence their performance. Leadership styles of both transformational and transactional types were chosen for examination. It was decided to focus on these leadership styles because of their prevalence.

## 2 Literature review

James MacGregor Burns introduced the concept of transactional leadership in 1978. Transactional leadership is a style in which leaders focus on the exchange of rewards and punishments to motivate and guide their followers in achieving specific goals. This leadership style emphasizes clear structures, expectations, and performance-based rewards. Transactional leaders do not work well in environments that promote innovation and creativity. Transformational leadership is often contrasted with transactional leadership. Self-motivated individuals who perform well in a structured and guided setting are necessary for transactional leadership.

The article "Comparative Analysis of Female Leadership Styles in Public and Private Sector Universities: A Study in Pakistan" was retracted in 2025. Reason: plagiarism.

The concept of transformational leadership was first introduced by James V. Downton in 1973. Transformational leadership is a leadership style characterized by inspiring and motivating followers to achieve their full potential and exceed their self-interests for the collective goals of the organization. Transformational leaders encourage creativity, innovation, and intellectual stimulation, thereby fostering a sense of empowerment and personal growth among their followers. In other words, transformational leadership chooses to influence rather than command people to inspire and encourage employees (Demirtas, 2020). Transactional leadership emphasizes the value of interactions between a supervisor and its employees [20]. This idea relies on the path-goal theory of incentives, which suggests that people are more likely to get things done if they are motivated to do so by progressing toward specific goals [21]. The transactional leader can inspire their team by determining what drives them and then providing it. This style of management is based on a barter system, in which employees' subservience is exchanged for financial rewards [22]. This style of leadership, which centers on the value of exchange, is appropriate only in certain cultural contexts. According to Ref. [23]; a transformative leader motivates followers through more than a simple moral example. Subordinates may develop their full potential and provide excellent results. As people perceive it, leadership is a process that affects its followers, raises the spirits of both the leader and the leader and is rooted in values and ideals [20]. According to Burns, transformational and transactional leadership are at different extremes on a continuum [22].

[23] argued that transformational and transactional styles of leadership are incompatible. Contrary to what you may have heard [24], stated otherwise: Instead, Bass argues that there is a mutual benefit between the two styles of leadership [25]. Bass classified leadership styles as transformative and transactional as complementary rather than mutually exclusive. In his "complete spectrum of leadership style " theory, a leader may effectively combine transactional and transformational approaches [26]. In addition [23], argued that any kind of change is beneficial. Alternatively, Bass (2018) argues that transformation may have both positive and negative effects. A transformational leader inspires followers to exceed their standards. Furthermore, they are moved to forego personal gains in favor of the collective [27]. By educating followers to adapt to new circumstances, boost their performance, and help the leader, team, and organization achieve their objectives, transformational leadership may also enhance transactional leadership. It improves morale and helps followers feel that their leader is making a difference [28]. The difference between transactional and transformational leadership is that the latter seeks to develop subordinates into future leaders, while the former seeks to maintain the status quo [26].

The article "Comparative Analysis of Female Leadership Styles in Public and Private Sector Universities: A Study in Pakistan" was retracted in 2025. Reason: plagiarism.

[29] found that female involvement in management positions has significant role in the finance and human talent departments, and that transactional and transformational leadership were the most appropriate for female leaders. Moreover, a moderate relationship between the type of leadership and female participation in management positions was also found.

[30] also advocate that female actual controlling shareholders of family companies could effectively suppress business violation. Furthermore, family emotional affection shows a role to moderate the relationship between female actual controlling shareholders and business violation. Kinship ties to family emotional, non-economic benefits are important reference points for business decision-making in family-owned businesses. Several studies have identified the following four dimensions of transformational leadership.

### 2.1 Transformational leadership dimensions

#### 2.1.1 Idealized influence

A transformational leader may exert an idealized impact by setting a personal example of dedication to the organization's objectives via charismatic role modeling. In doing so, the leader earns the esteem of his or her subordinates and the confidence of those who follow [31]. Transformational leaders display such behavior, which makes them role models for subordinates [22]. These leaders are respected, acknowledged, and trusted because of their expertise, perseverance, and resolution [32]. They prioritize the needs of subordinates above their own, create and uphold higher moral and ethical standards, take calculated risks, and do not abuse their position of power [33]. These leaders are also regarded as good decision-makers and effective communicators of the organization's vision and purpose [20]. Because of these leadership behavioral traits, followers emulate these leaders and want to be like them. This dimension contains two conceptually separate components: the first is "idealized influence behavior,” which is tied to the leader's behavioral traits, and the second is "idealized influence ascribed,” which is linked to the traits that the leader's subordinates attribute to them [34]. The likelihood that followers will internalize and attain the conveyed objectives is higher when charismatic leaders have faith in their subordinates to do so [35].

The article "Comparative Analysis of Female Leadership Styles in Public and Private Sector Universities: A Study in Pakistan" was retracted in 2025. Reason: plagiarism.

#### 2.1.2 Inspirational motivation

Inspirational motivation is a leader's capacity to motivate and inspire people. Transformational leaders must establish a clear vision of the future, explain group expectations, and commit to set objectives. Transformational leaders must express their messages accurately, with strength, and authority. Other crucial leadership traits include optimism, excitement, and positivity [31]. According to Naguni et al. (2006), inspirational motivation is the quality of charismatic leadership in which leaders arouse their followers' ambitions by making emotional appeals to them and offering enticing predictions of the future [20]. These people inspire the group's spirit, set clear expectations that their followers are prepared to meet and show a commitment to the group's goals and vision [34]. A leader who inspires followers is seen as knowledgeable, enlightened, and attentive to challenges; requires no trusting cooperation from followers; and increases the commands of followers by assisting them in achieving the set objectives [35].

[36] proposed that servant leadership is positively connected to employees' intrinsic motivation and service innovative behavior. Moreover, employees' intrinsic motivation partially mediates the link between servant leadership and their service innovative behavior. Additionally, employees’ identification with the leader not only moderates the association between servant leadership and their intrinsic motivation, but also controls the mediating role of intrinsic motivation, in such ways that these two effects are more clear among the workforces with higher levels of identification with the leader than lower ones.

#### 2.1.3 Intellectual stimulation

Transformational leaders push their subordinates to be more innovative and creative by asking them questions and thinking critically about what they are doing. This kind of leadership also encourages followers to question their beliefs and morals, as well as those of the leader and organization. In addition, finding a solution is performed in a way that involves everyone. Followers' creative ideas are welcomed, even if they go against what the leader thinks. It is good when subordinates take different approaches to problems and solve them in their way [20,33]. Transformational leaders are encouraged to think independently and creatively: A good leader encourages his team to go outside the box when coming up with ideas, and he does this by including them in decision-making. Transformative leaders encourage followers to think critically and provide their ideas. A good leader influences people to reframe situations in a new way. Leaders inspire their teams to be great by sharing their vision of the future [37].

The article "Comparative Analysis of Female Leadership Styles in Public and Private Sector Universities: A Study in Pakistan" was retracted in 2025. Reason: plagiarism.

#### 2.1.4 Individualized consideration

There are individual wants and requirements among the members of each organization. Some people, for instance, are driven by financial incentives, while others seek novel experiences. Therefore, transformative leaders pay attention to details and cater to each person's specific requirements. The leader needs eavesdropping and observing skills to determine what drives each team member. The transformative leader creates an opportunity for individualized training for each team member via one-on-one coaching and mentoring. By participating in these events, team members are allowed to learn, develop, and enjoy their work [37]. A transformational leader acts as a mentor and cares about subordinates' success and growth to the highest level (Avolio, 1999) [26]. say that a leader must develop himself or herself if he or she wants to help his or her followers grow. Here, the leader shows that he or she understands that each follower has different needs and goals by acting differently around different people [33]. The leader makes it easy for followers to learn and grow by maintaining two-way communication, tailoring their interactions with subordinates, listening to them carefully, and giving them tasks with ongoing evaluations and support if needed [33]. Consideration behavior is essential for both transformational and transactional leadership [24]. (Seltzer & Bass, 1987). There is much evidence from different organizations and cultures that transformational leaders are more effective than transactional leaders because of these traits [26].

### 2.2 Transactional leadership dimensions

Three dimensions of transactional leadership and "non-leadership behavior have been discussed in the literature [32,38]; Bass &Avolio, 1994; [39]. These four factors are exchanged on different levels between the leader and the people who follow them [24]. Here, unlike a transformational leader, neither the need nor the growth of subordinates is a focus. However, similar to transformational leadership, transactional leadership has an ethical aspect. [40]; p. 185) say that "the moral legitimacy of transactional leadership is demanding in many ways. It depends on giving others the same freedom and chances you want for yourself, telling the truth, keeping promises, giving everyone what they deserve, and using good incentives or punishments".

The article "Comparative Analysis of Female Leadership Styles in Public and Private Sector Universities: A Study in Pakistan" was retracted in 2025. Reason: plagiarism.

#### 2.2.1 Contingent reward

Recognition and prizes for achieving objectives are used by transactional contingent reward leadership as motivational factors for members. Through transformational leadership, an organization's members become more personally and socially connected to leaders and the group's purpose and objectives (Demirtas, 2020). In this model, an exchange occurs between leaders and subordinates. In exchange for obedience and work, subordinates receive a certain amount of money [20]. The transactional leader deals with subordinates that outline the goals to be reached and the rewards for doing so. Once the goals are reached, the leader gives agreed-upon rewards (Naguni et al., 2006). Peters and Waterman (1982) stated that contingent rewards are an excellent way to give subordinates positive feedback and to make them happy. However, many studies show that contingent rewards are not as effective as other types of transformational leadership in terms of subordinates' satisfaction, performance, and growth [33]. However, the meaning of leadership practices depends on the cultural and organizational contexts in which they are used. Ingroup collectivism, on the other hand, looks at how attached, loyal, and devoted people are to their organizations and families, and how willing they are to make sacrifices for them [41]. Some countries, like Iran, Philippines, Malaysia, Indonesia, Thailand, and India, are high in "humane orientation” and "ingroup collectivism,” which means that people have strong bonds, loyalty, and care for their families, institutions, and communities. In these countries, people would instead be thanked by their leaders and coworkers rather than get paid for the extra help or time they have given the institution [41]. Humane orientation is the degree to which a society or culture encourages people to be fair, selfless, generous, helpful, considerate, and sensitive to others [41].

#### 2.2.2 Management-by-exception (active)

This is a more proactive and successful kind of transactional leadership that corrects behavior by looking for what was done incorrectly rather than what was done well. As in "micromanagement,” the leader carefully checks job performance for faults to address issues before they arise (Demirtas, 2020). This kind of leader pays close attention to their team's progress, keeps track of errors and deviations from the norm, and intervenes as necessary [20,40]. A passive kind of management known as "management by exception” A leader who uses management by exception waits for problems to escalate before taking action, may be unaware of problems until they are brought to their attention by subordinates, and is therefore unlikely to achieve desired results [33,40]. Both kinds of management by exception are less effective than the traditional types of leadership, yet they are sometimes necessary [42].

The article "Comparative Analysis of Female Leadership Styles in Public and Private Sector Universities: A Study in Pakistan" was retracted in 2025. Reason: plagiarism.

The beliefs, culture, and behavioral patterns of a society will ultimately determine whether or not its members adopt any of these leadership styles. Academics in Thailand were studied by Dastoor, Suwant Tochin, and Golding (2013), who analyzed the connection between leadership styles and work satisfaction. They were able to do this by drawing from both the transformational and transactional models of leadership. Faculty job satisfaction seems to be more strongly related to a leader's transformative rather than transactional approach, according to the data. According to Ref. [21]; who conducted similar research at a university in the Midwest of the United States using the same leadership approach, transformational leadership behaviors have a strong correlation with faculty satisfaction, while transactional leadership behaviors have a weak correlation.

The expected value that a leader delivers to the organization of the discrete behavioral events that occur over a typical period can define a leader's job performance [43]. It may also be described as the effectiveness with which leaders carry out their responsibilities (Torlak & Kuzek, 2019), and it is often assessed using many metrics (Pradhan & Jena 2017; [44]. Leaders' performance often depends on the knowledge, ability, competence, and behavior required to accomplish the position [45]. The majority of businesses place a high value on employee job performance since it is crucial to establishing a long-term competitive advantage. Even in the same society, the way these leadership styles are used and how big they are could be different in different situations. For example, in contrast to Refs. [21,46] used the same leadership theory paradigm to look at a similar relationship at a university in North Carolina, United States, in an informal educational setting. Stump found that the transformational leadership style was strongly linked to the job satisfaction of faculty members. Also, the first dimension of the transactional leadership style, contingent reward, had a stronger positive relationship with faculty job satisfaction than the second dimension of the same style, management-by-exception (active). On the other hand, the last dimension of this style.

#### 2.2.3 Management-by-exception (passive)

This is a little more successful kind of corrective transactional leadership behavior in which the leader focuses on errors only after they have taken place and then applies solutions to the issues. Before taking any kind of action, the leader waits for something to go wrong (Demirtas, 2020 & [47]. It had a significant negative relationship with faculty job satisfaction. The above shreds of evidence show that leadership styles are rooted in situations. Many recently completed studies show that transformational and transactional leadership styles are well known, accepted widely, and are becoming topics of interest to scholars who study organizational success, employee performance, and organizational development, among other things [3]; Rehman et al., 2012). Along with studying both leadership styles, many studies have found an association between transformational and transactional leadership and employee job performance. Both leadership styles are positively associated with employee job performance [[3], [4], [5]].

The article "Comparative Analysis of Female Leadership Styles in Public and Private Sector Universities: A Study in Pakistan" was retracted in 2025. Reason: plagiarism.

Therefore, based on the literature review the researcher proposed the following hypotheses to compare transformational, transactional leadership and job performance perceived by female university leaders working in the public and private sector universities of Pakistan.

### 2.3 Objectives/hypotheses

H1 There is a statistically significant difference in the leadership style of female leaders in public and private sector universities

H2 There is a statistically significant difference in the job performance of female leaders of public and private sector universities

H3 There is a statistically significant difference in the transformational and transactional leadership style of the female leaders working at different positions in public and private sector universities

H4 There is a statistically significant difference in the perceptions of female leaders towards their job performance working at different positions in public and private sector universities

## 3 Data and methodology

This study used a mixed-method research design (Fig. 1). In this method, the quantitative data were collected in the first phase, while qualitative data were collected in the second phase. Two research instruments, an adopted questionnaire, and a self-developed interview schedule, were used for data collection. In this study we used mixed methods due to the following reasons: first, to collect both quantitative and qualitative data, which can provide a more comprehensive understanding. Secondly, in this study, we used qualitative data to explore and explain the results of quantitative data. The mixed method helped to provide a deeper understanding of the findings and their implications, which can make research more relevant and impactful to a wider audience. Overall, mixed methods research can be a valuable tool for researchers to gain a deeper and more comprehensive understanding of research. The Likert-based questionnaire had 33 statements and three sections. The first two sections were related to transformational and transactional leadership style, which was adopted from Ref. [48] *MLQ Multifactor Leadership Questionnaire*. The third section was related to job performance, which the researchers developed. Similarly, in a semi-structured interview schedule, there were seven questions. All deans, HODs, directors, Senior Faculty, and coordinators belonged to the female gender working in public and private sector universities in Punjab Province of Pakistan formed the population. Pakistan is a patriarchal society, and women face many challenges in achieving leadership positions. Therefore, it is important to understand the specific experiences of female leaders in Pakistan to develop effective strategies for increasing their representation in leadership positions. The following are the major reasons to choose females in our research. First, according to a 2021 report by the American Council on Education, women make up only 30 % of presidents of four-year colleges and universities in the United States. This means that there is a need to understand the experiences and challenges of female university leaders to increase their representation in these positions. Second, studies have shown that universities with more female leaders tend to have more inclusive and supportive cultures for all students. This is because female leaders are often more likely to be approachable and empathetic, and they are more likely to create policies and practices that benefit all students. Third, seeing female leaders in positions of power can inspire and motivate female students to pursue their own leadership goals. This is especially important in STEM fields, where women are still underrepresented.

The article "Comparative Analysis of Female Leadership Styles in Public and Private Sector Universities: A Study in Pakistan" was retracted in 2025. Reason: plagiarism.

From the said population, a sample of 200 females from 10 universities (five public & five private) was selected through purposive and simple random sampling techniques. Before the application of the instruments, their validity and reliability were confirmed by seeking expert opinions and conducting pilot testing (with 50 responded data) on a small sample. The reliability of the quantitative instrument occurred as (α = 0.87). Later, the researchers collected the data personally and through the online method using Google Forms. SPSS was used to analyze quantitative data, while the thematic approach was used to analyze qualitative data.

Simple statistics are a valuable tool for researchers because they are relatively easy to understand and interpret. They can also be used to test a wide variety of hypotheses. In the context of the hypotheses listed above, simple statistics can provide valuable insights into the leadership styles, job performance, and perceptions of female leaders in public and private sector universities. In addition to these reasons, there are a few other reasons why it is important to rely on simple statistics to support the analysis of the hypotheses. First, simple statistics are relatively inexpensive to collect and analyze. This is important for researchers who are working with limited resources. Second, simple statistics are relatively easy to communicate to a wide audience. This is important for researchers who want to share their findings with policymakers, practitioners, and the general public. There are also some limitations to using simple statistics. For example, simple statistics can only be used to test hypotheses about the mean or median of a population. This means that they cannot be used to test hypotheses about the distribution of a population. Additionally, simple statistics can be sensitive to outliers, which can distort the results of a study. Despite these limitations, simple statistics are a valuable tool for researchers who are interested in testing hypotheses about female leadership in public and private sector universities. They are relatively easy to understand, interpret, and communicate, and they can be used to test a wide variety of hypotheses.

Based on both analyses, the following results are recorded.

Fig. 1 The mixed-method study design.

**Fig. 1:** Study design.

## 4 Quantitative findings

H_1_: There is a statistically significant difference in the leadership style of the female leaders of public and private universities.

## 5 Qualitative findings

The qualitative data were collected from the ten female leaders working in public and private sector universities. After analyzing and interpreting quantitative data, the researcher used the semi-structured interview technique. Later, the data collected in interviews were converted into themes, and a thematic technique was adopted to interpret the qualitative data to corroborate the results of quantitative data. The complete interpretation of qualitative data is presented below.

### 5.1 Theme A: awareness

Q.1. what do you know about the transformational leadership style?

In response to this question, RF1 stated, "People using transformational leadership always inspire their employees through various tactics such as encouraging, inspiring, and motivating them to increase their performance. RF2 responded "It is something passionate and enthusiastic leadership”. RF3 answered, "Transformation means a characteristic patron of interaction among the most active participation in any activity, which appears that one system has replaced another. It is an essential process that brings changes and transforms people. Transformation leadership is concerned with emotions, values, ethics, standards, and long-term goals that include assessing the followers' motives, satisfying their needs, and treating them as full human beings. It incorporates charismatic and visionary leadership, and though the leader plays a pivotal role in precipitation change, followers and leaders are inextricably bound together in the transformation process”. RF4 said that "it can be considered as inspiration in which people present themselves as a role model”. RF5 explained that "It is a style which can inspire people towards positive changes. It focuses on the positive role of supervision through helping and guiding every team member”. RF6 said, "People with this leadership style are known as a supporter and good guides. They help their team members achieve their firm's common goals”. RF7 described that this style of leadership brings positive changes in employees, which are essential for the success of a transformational leader”. RF8 and RF9 said, "This leadership style involves other workers participating in important tasks”. RF10 voiced that in this leadership, leaders motivate, inspire, and encourage their workers to achieve the firm's goals. This style is very helpful for the success of any organization. Based on the above qualitative data, it has been revealed that all respondents have a good awareness of the transformational leadership style.

The article "Comparative Analysis of Female Leadership Styles in Public and Private Sector Universities: A Study in Pakistan" was retracted in 2025. Reason: plagiarism.

### 5.2 Theme B: awareness

Q.2. what do you know about the Transactional leadership style??

In reply to this question, RF1, RF2, and RF3 stated, "Transactional style of a leader deals with their followers by offering various types of rewards and punishments. These leaders use these strategies to catch the attention of their employees. This is a very hard leadership style and most men use this style when employees fail to achieve any goal these leaders have to deal with that employee with an iron hand. RF4 stated that the "Transactional style focuses towards leading by making good plans and offering benefits for workers to achieve the targets of the firm”. RF5 described that "Transactional leadership style focuses on the role of the organization on group performance. It also uses punishment and rewards system to improve employee performance”. RF6 responded, "People using this style are known as hard leaders. They use punishment and rewards model on the employees to achieve the targets of their company”. RF7 answered that "Transactional type of leaders use penalty and rewards system on the employees to achieve the goals of their organization as well as to enhance their job performance”. RF8 replied "This is a leadership style which does not involve other people to participate. It works on a governing system. Leaders practicing transactional style motivate workers by announcing rewards on good performance and punishment on poor performance”. RF9 said that the "leadership style of transactional is that in which leaders attract workers through rewards and punishment to achieve their company's goals. RF10 voiced that the "Transactional leadership style focuses on the importance of supervision, structure, and teamwork. Leaders who employ this approach concentrate on specific tasks and provide incentives and penalties to inspire their followers”. Because of the said claims of the respondents RF1 to RF10, it has been discovered that the majority of the participants have a clear awareness of the transactional leadership style.

The article "Comparative Analysis of Female Leadership Styles in Public and Private Sector Universities: A Study in Pakistan" was retracted in 2025. Reason: plagiarism.

### 5.3 Theme C: practices

Q.3. Which leadership style you are practicing in your university? why?

In response to this question, the responses of RF1 to RF10 were mentioned below: RF1 responded, "I practice transformational leadership style as I believe in teamwork, creating a positive work environment in my organization”. RF2 stated, "I am using transactional leadership because people are motivated by incentives”. RF3 answered, "Both leadership styles are being pursued in my university, and a blend is being implemented. Both are appropriate in one way or another, and this blended form fulfills many needs. One requires charismatic leadership, while the other provides good management ideas and gives workers what they desire in exchange for attaining what leaders desire. It assumes that employees are not self-motivated and need structure, instruction, and monitoring to complete tasks appropriately and on time. So, according to my opinions, I favor practicing transactional leadership style”. RF4 replied that "both together styles work according to the situation and both work nicely. I like to use transformational style as it focuses on team building and change inside the organization”. RF5 responded that "I prefer to use transactional leadership in my university, as I consider that every member in a team is essential for the progress of a university”. RF6 stated that "I practice to use the transformational style of leadership because it is the need of time to work all together for the progress of university through teamwork”. RF7 voiced that "I prefer to use transformational style. It is a more flexible style to improve performance as well as to achieve targets”. RF8 explained that "According to the situation, both leadership styles are important for me; I use both styles in my university”. RF9 described that "I often try to practice transformational leadership as the university is a place where people are encouraged instead of rewards and punishment to work for the common goals of the university which is standard and quality of education”. Moreover, being female I have to work with my subordinate and colleagues based on democracy instead of dictatorial. RF10 replied that "I practice transformational leadership style in my university because this style focuses on change”. So based on the claims of the female leaders, it has been revealed that respondents RF2, RF3, RF5, and RF8 prefer to use a transactional leadership style in their universities, while respondents RF1, RF4, RF6, RF7, RF9, and RF10 stated that they practice transformational style of leadership in the organizations.

The article "Comparative Analysis of Female Leadership Styles in Public and Private Sector Universities: A Study in Pakistan" was retracted in 2025. Reason: plagiarism.

### 5.4 Theme D: awareness

Q.4. How do you perceive Job Performance?

In reaction to this question, the following explanations of the respondents from RF1 to RF10 are presented**:** RF1 said that "According to my point of view when you introduce new techniques to enhance your creative skills compete with the words what going on all over the world in the fields of education you adopt or create your style and listen to your subordinates respect their ideas, and on the bases of all you get better and better ways of work and in the end its converts in better job performance”. RF2 explained that "Job performance is the creative work with innovation and introducing new ideas instead of old ideas”. RF3 told that "Job performance can be described as the competence to transform innovation inputs into outputs, and in this way, the ability to transform innovation capability and effort into market implementation, is its requirement. Sometimes, the outcome of job performance is innovation-oriented success at any place”. RF4 voiced that "Innovative performance is like implementing new ideas inside university”. RF5 responded that "Innovative performance is the use of an idea or creativity to improve the products, process that increases the performance of products”. RF6 described that "Creating novel things in job place is an innovative performance”. RF7 explained that "People can input new ideas, a concept in their outputs. Such as involvement of technological tools to achieve the innovative performance at the workplace”. RF8 replied that "Creating novelty, introducing new things or ideas in any product or a new idea is considered innovative performance”. RF9 responded that "It is a new idea in performance such as new product, etc.”. RF10 highlighted that "The creation and use of a new idea, concept, or product or services to increase the innovative performance in a company is an innovative performance”. Given the statements of the participants, it has been discovered that the majority of the female leaders have a good and clear awareness of innovation and innovative job performance.

The article "Comparative Analysis of Female Leadership Styles in Public and Private Sector Universities: A Study in Pakistan" was retracted in 2025. Reason: plagiarism.

### 5.5 Theme E: transformational leadership and job performance

Q5: How the transformational leadership styles increase job performance?

Responding to this question, respondent RF1 explained, that the transformational style impacts better performance because, in this style, most leaders motivate their workers to achieve the firm's goals. RF2 said, "Leaders using transformational style develop a strong social bond and affect employee performance. These leaders increase the emotional connection between followers and leader in a way that employee feels confidence and struggle to achieve the firms' goals”. RF3 voiced that “Transformational leaders' emphasis on creative aspects takes to improvement in the projects' innovation performance”. RF4 voiced that "Transformational leaders should be well prepared to deliver lectures and to answer the questions of students as well as to increase their performance”. RF5 answered that "Transformational leaders can achieve better performance through giving positive working environment”. RF6 told that "Being team leader, the transformational leader can increase their job performance by involving members in the success of their novel ideas”. RF7 stated that "These leaders develop positive relations among employee and create a healthy environment inside the organization and motivate employees to work for the betterment of their organization”. RF8 responded, "Without a good team, it is impossible to win the match. So, transformational leaders develop a strong team formation that the basic purpose of this leadership style can increase job performance”. RF9 said, "Exercising transformational leadership style can improve job performance through motivation, etc.”. RF10 voiced that "This style focuses on the motivation of the followers. This motivation enables followers to work towards innovation which increases the job performance of the leaders. Moreover, he said that there is no style for all situations; I change my style considering the nature of the situation as sometimes I have to use an iron hand instead of motivation for completing a task through subordinates”. Given the mentioned claims of the female leaders, it has been exposed that most of the participants of this study agreed that there is a significant influence of transformational leadership style on the job performance of the female leaders.

### 5.6 Theme F: transactional leadership and job performance

Q6: How the transactional leadership styles increase job performance?

The article "Comparative Analysis of Female Leadership Styles in Public and Private Sector Universities: A Study in Pakistan" was retracted in 2025. Reason: plagiarism.

In feedback to these questions, the important claims of the respondents are demonstrated as under: RF1 claimed that the "Transaction process between leaders and workers directed to display a satisfactory performance. Leaders using transactional style motivate followers by announcing incentives to increase their performance instead of creating self-motivation, self-commitment and self-interest of the employees towards company goals”. RF2 responded that "Because the use of rewards and punishment model automatically increases the performance of human beings”. RF3 stated that "Transactional leadership is like managers that give employees something they want in exchange for their needs. It posits that workers are not self-motivated and require structure, instruction, and monitoring to complete tasks correctly. All this enhances their job performance. Transactional leadership is likely beneficial during a crisis or in projects requiring linear and particular procedures. This type is also beneficial for large companies for general administration”. RF4 voiced that "transactional leaders create a good thinking and achieve company target by introducing rewards and punishment system to motivate followers to work appropriately”. RF5 answered, "By watching the rewards and punishments to motivate followers”. RF6 described that "It is also a significant leadership style and through punishment and rewards system only performance can be increased instead of better job performance. Innovation can only and only when a person thinks freely on any idea”. RF7 said, "This type of leader is rigorous, and they also use rewards and punishment model to increase an employee's performance, which affects their performance ". RF8 & RF9 voiced that "Some people use this type of leadership, it is also useful for lower-level organization and through it, and these organizations improve their job performance to some extent”. These leaders give rewards to their employees and in this way, they motivate people to perform well”. In the light of stated claims of the female leaders, most female leaders claimed that transactional leaders use rewards and punishment systems to motivate their subordinates to achieve the organization's targets. In this way, this leadership style had a significant role in job performance.

### 5.7 Theme F: quality

Q7: How can you enhance the quality of education at your institution?

In response to this question, RF1 said that "quality of education can be enhanced by using new teaching techniques, introducing new assessment techniques, and using social media for better teaching-learning can promote creative skills”. RF2 voiced that the "quality of education can be increased by continuously watching and implementing educational policies”. RF3 responded, "By applying both types of leadership as these are alternatives of each other. The goal of engaging with others in this sort is to create a bond that boosts motivation and morality in both leaders and followers”. RF4 stated, "It needs to motivate students, to be honest with their studies. Lectures should be prepared well to implement transformational leadership. Involve students in lectures. Ask again and again questions … answer them. Sometimes prizes work well”. RF5 stated that "at university level quality of education can be increased only through research and by studying more books and literature”. RF6 voiced that "Quality of education can be improved by the fair implementation of educational policies in true spirit”. RF7 answered, "I think that by using transformational leadership style, we can improve the quality of education by providing a positive working climate inside the organizations”. RF8 replied, "By giving proper training to the teachers, quality of education can be improved”. RF9 responded that "by executing fair and promote policies and providing academic culture, and providing appreciation, and rewards to the teacher quality of education can be achieved”. RF10 described that "quality of education can be enhanced by proving rewards to the teachers for implementation of policies”. Given the said statements of the respondents, it has been established that all the respondents agreed that the quality of education could be improved by observing educational policies and implementing these policies fairly, and motiving teachers and students in the whole learning process by providing conducive teaching and learning environment and by giving incentives.

The article "Comparative Analysis of Female Leadership Styles in Public and Private Sector Universities: A Study in Pakistan" was retracted in 2025. Reason: plagiarism.

### 5.8 Summary of qualitative findings

**Table:** 

Theme	Question	Response
Awareness	What do you know about the transformational leadership style?	All respondents have a good awareness of the transformational leadership style
	What do you know about the Transactional leadership style??	The majority of the participants have a clear awareness of the transactional leadership style.
	How do you perceive Job Performance?	Majority of the female leaders have a good and clear awareness of innovation and innovative job performance
Practices	Which leadership style you are practicing at your university? Why?	6 respondents out of 10 stated that they practice a transformational style of leadership in the organizations because this style focuses on change
Transformational Leadership and Job performance	How the transformational leadership styles increase job performance?	Participants of this study agreed that there had a significant influence of transformational leadership style on the job performance of female leaders.
Transactional leadership and Job performance	How the transactional leadership styles increase job performance?	Female leaders claimed that transactional leaders use rewards and punishment systems to motivate their subordinates to achieve the organization's targets. In this way, this leadership style had a significant role in job performance.
Quality	How can you enhance the quality of education at your institution?	The quality of education could be improved by observing educational policies implementing these policies fairly, and motivating teachers and students in the whole learning process by providing a conducive teaching and learning environment and by giving incentives.

In summary, it has been revealed that most interviewees had a solid understanding of the transformational leadership approach. According to the findings, the majority of interviewees had a firm grasp of the transactional leadership style. According to the findings, the majority of female leaders are practicing a transformational leadership style. In contrast, few female leaders practice transactional leadership in public and private universities. The majority of the female leaders had a firm grasp of what innovation is and how job performance is achieved. The majority of the female leaders believed that the transformational leadership style significantly affected their ability to innovate. The majority of the females stated that transactional leaders employ reward and punishment systems to drive their subordinates to achieve academic objectives, which also significantly affects creative output. This research has established that most female leaders believe that the quality of education could be improved by observing educational policies and fairly implementing these policies and by motivating teachers and students throughout the entire learning process by creating a positive learning environment and offering incentives.

### 5.9 Summary of overall findings

**Table:** 

Hypotheses	Acceptance/Rejection
**H**_**1**_**:** There is a statistically significant difference in the leadership style of female leaders in public and private sector universities	Accepted
**H**_**2**_**:** There is a statistically significant difference in the job performance of female leaders of public and private sector universities	Accepted
**H**_**3**_**:** There is a statistically significant difference in the transformational and transactional leadership style of the female leaders working at different positions in public and private sector universities	Accepted
**H**_**4**_**:** There is a statistically significant difference in the perceptions of female leaders towards their job performance working at different positions in public and private sector universities	Accepted

Table 1 shows the results of *t*-test statistics. Results show statistically significant differences between the leadership styles of females of public and private sector universities regarding transformational leadership style, transactional leadership style, and their performance. It is noticeable from the results that female leaders working in public sector universities had a higher mean and standard deviation (M = 3.96, SD = 0.519) while female leaders working in private sector universities had a lower mean and standard deviation (M = 3.55, SD = 0.587) regarding transformational leadership style. The calculated p-value (0.000 <0 .05 levels) also acknowledged significant differences between female leaders of public and private sector universities regarding transformational leadership style. It is evident from the outcomes that female leaders of public sector universities had a higher mean and standard deviation (M = 3.38, SD = 0.758) while female leaders working in private sector universities had a lower mean and standard deviation (M = 2.94, SD = 0.602) regarding transactional leadership style. The computed p-value (0.000 <0 .05 levels) also acknowledged significant differences between public and private sector university female leaders regarding transactional leadership style. It is apparent from the outcomes that female leaders of public sector universities had a higher mean and standard deviation (M = 4.10, SD = 0.482) while female leaders working in private sector universities had a lower mean and standard deviation (M = 3.95, SD = 0.434) regarding job performance. The computed p-value (0.016 <0 .05 levels) also acknowledged that there were significant differences between female leaders of public and private sector universities regarding job performance. Fig. 2 shows the graphical representation of sector-wise comparisons of transformational, transactional leadership and performance of female leaders in universities.

The article "Comparative Analysis of Female Leadership Styles in Public and Private Sector Universities: A Study in Pakistan" was retracted in 2025. Reason: plagiarism.

**Table 1:** University sector-wise comparisons of females' transformational and transactional leadership styles (*N* = 200).

Variables	University Sector	N	Mean	Std. Deviation	t-value	p-value
Transformational	Public	110	3.96	.519		
	Private	90	3.55	.587	5.173***	.000
Transactional	Public	110	3.38	.758		
	Private	90	2.94	.602	4.621***	.000
Performance	Public	110	4.10	.482		
	Private	90	3.95	.434	2.430***	.016

*p < 0.05, **p < 0.01, ***p < 0.001.

**Fig. 2:** University-sector-wise comparisons of transformational, transactional leadership and performance of female leaders.

Based on the above results, it has been revealed that female leaders working in public sector universities had a higher attitude toward practicing transformational leadership, transactional leadership, and job performance. While female leaders working in private sector universities had a lower attitude towards practicing transformational & transactional leadership styles and job performance. Therefore, both research hypotheses (a) H1: There is a statistically significant difference in the transformational and transactional leadership style of the female leaders in public and private sector universities, and (b) H2: There is a statistically significant difference in the job performance of female leaders of public and private sector universities are accepted.

Table 2 shows that one-way ANOVA was used to explore position-wise differences in female leaders regarding transformational leadership style. Results discovered statistically insignificant differences among groups as demonstrated by one-way ANOVA (F (5,194) = 1.970, p = 0.085 >0 .05). Based on said results, it has been revealed that female leaders working in all positions had an equal attitude towards practicing transformational leadership style in their universities. Thus, the research hypothesis (c) H1: There is a statistically significant difference in the transformational leadership style of the female leaders working at different positions in public and private sector universities is rejected.

**Table 2:** Position-wise comparisons of transformational leadership style practiced by female leaders in public and private sector universities (*N* = 200).

	Sum of Squares	df	Mean Square	F	Sig.
Between Groups	3.311	5	.662	1.970	.085
Within Groups	65.213	194	.336		
Total	68.524	199			

Table 3 shows the position-wise mean differences in female leaders practicing transformational leadership styles in their universities. According to the mean value of all positions, there was a little bit of difference among female leaders regarding practicing transformational leadership styles such as Dean (M = 3.5417), HOD (M = 3.6556), Director (M = 3.7240), Senior Faculty (M = 3.7864), Coordinator (M = 3.7500), and Others (M = 4.1042).

**Table 3:** Position-wise Mean Score & Std. Deviation of female leaders practicing transformational leadership style (N = 200).

Positions	N	Mean	Std. Deviation	Std. Error	95 % Confidence Interval for Mean	
					Lower Bound	Upper Bound
Dean	12	3.5417	.47073	.13589	3.2426	3.8408
HOD	30	3.6556	.58343	.10652	3.4377	3.8734
Director	16	3.7240	.58192	.14548	3.4139	4.0340
Senior Faculty	110	3.7864	.54878	.05232	3.6827	3.8901
Coordinator	12	3.7500	.75962	.21928	3.2674	4.2326
Other	20	4.1042	.67477	.15088	3.7884	4.4200
Total	200	3.7767	.58681	.04149	3.6948	3.8585

Results demonstrated in Table 4 describe that one-way ANOVA was used to explore position-wise differences in female leaders regarding transactional leadership style. Results exposed statistically insignificant differences among groups as demonstrated by one-way ANOVA (F (5,194) = 2.189, p = 0.057 >0 .05). Given said outcomes, it has been discovered that female leaders in all positions had an equal attitude towards practicing transactional leadership style in their universities. Thus, the research hypothesis (c) H1: There is a statistically significant difference in the transactional leadership style of the female leaders working at different positions in public and private sector universities is rejected.

The article "Comparative Analysis of Female Leadership Styles in Public and Private Sector Universities: A Study in Pakistan" was retracted in 2025. Reason: plagiarism.

**Table 4:** Position-wise comparisons of transactional leadership style practiced by female leaders in public and private sector universities (*N* = 200).

	Sum of Squares	df	Mean Square	F	Sig.
Between Groups	5.590	5	1.118	2.189*	.057
Within Groups	99.097	194	.511		
Total	104.688	199			

*p < 0.05, **p < 0.01, ***p < 0.001.

Table 5 shows the position-wise mean differences in female leaders practicing transactional leadership style in their universities. According to the mean value of all positions, there was a little bit of difference among female leaders regarding practicing transactional leadership styles such as Dean (M = 3.0521), HOD (M = 3.1833), Director (M = 3.2969), Senior Faculty (M = 3.1182), Coordinator (M = 3.0417), and Others (M = 3.6563).

**Table 5:** Position-wise Mean Score & Std. Deviation of female leaders practicing transactional leadership style (N = 200).

Positions	N	Mean	Std. Deviation	Std. Error	95 % Confidence Interval for Mean	
					Lower Bound	Upper Bound
Dean	12	3.0521	.73171	.21123	2.5872	3.5170
HOD	30	3.1833	.86274	.15751	2.8612	3.5055
Director	16	3.2969	.74983	.18746	2.8973	3.6964
Senior Faculty	110	3.1182	.66529	.06343	2.9925	3.2439
Coordinator	12	3.0417	.77484	.22368	2.5494	3.5340
Other	20	3.6563	.66252	.14815	3.3462	3.9663
Total	200	3.1875	.72531	.05129	3.0864	3.2886

Table 6 shows that one-way ANOVA was used to explore position-wise differences in female leaders regarding job performance. Results informed statistically insignificant differences among groups as revealed by one-way ANOVA (F (5,194) = 0.910, p = 0.476 >0 .05). According to the said results, it has been exposed that female leaders working in all positions had an equal attitude towards job performance. Thus, the research hypothesis (d) H1: There is a statistically significant difference in the perceptions of female leaders towards job performance working at different positions in public and private sector universities is rejected.

The article "Comparative Analysis of Female Leadership Styles in Public and Private Sector Universities: A Study in Pakistan" was retracted in 2025. Reason: plagiarism.

**Table 6:** Position-wise comparisons of job performance of female leaders in public and private sector universities (*N* = 200).

	Sum of Squares	df	Mean Square	F	Sig.
Between Groups	.993	5	.199	.910	.476
Within Groups	42.368	194	.218		
Total	43.361	199			

*p < 0.05, **p < 0.01, ***p < 0.001.

Table 7 shows the position-wise differences in female leaders’ perceptions of their job performance. According to the mean value of all positions, there was a little bit of difference among female leaders such as Dean (M = 4.0449), HOD (M = 4.0667), Director (M = 4.0433), Senior Faculty (M = 4.0112), Coordinator (M = 4.3013), and others (M = 3.9846).

**Table 7:** Position-wise Mean Score & Std. Deviation of female leaders regarding job performance (N = 200).

Positions	N	Mean	Std. Deviation	Std. Error	95 % Confidence Interval for Mean	
					Lower Bound	Upper Bound
Dean	12	4.0449	.29785	.08598	3.8556	4.2341
HOD	30	4.0667	.43078	.07865	3.9058	4.2275
Director	16	4.0433	.58983	.14746	3.7290	4.3576
Senior Faculty	110	4.0112	.42770	.04078	3.9304	4.0920
Coordinator	12	4.3013	.57232	.16521	3.9376	4.6649
Other	20	3.9846	.61771	.13812	3.6955	4.2737
Total	200	4.0388	.46679	.03301	3.9738	4.1039

## 6 Discussion

The findings of this study reveal notable differences between female leaders in public sector universities and private sector universities regarding their leadership styles and perceptions towards job performance. Specifically, female leaders in public sector universities exhibited a higher level of attitudes towards practicing both transformational and transactional leadership styles compared to their counterparts in private sector universities. The higher level of attitudes towards practicing transformational leadership style among female leaders in public sector universities suggests that they are more likely to inspire and motivate their followers, promote intellectual stimulation, and foster a sense of empowerment and personal growth. This finding aligns with the nature of public sector universities, where there may be a greater emphasis on social impact and community development.

Furthermore, the higher level of attitudes towards practicing transactional leadership style among female leaders in public sector universities suggests a focus on clear structures, expectations, and performance-based rewards. This may be attributed to the bureaucratic nature of public sector institutions, where processes, rules, and regulations play a significant role in decision-making and resource allocation. On the other hand, female leaders in private sector universities demonstrated a moderate level of attitude toward practicing both transformational and transactional leadership styles. This may be indicative of the unique characteristics and dynamics present in private-sector universities, which may prioritize efficiency, competitiveness, and business-oriented approaches.

The article "Comparative Analysis of Female Leadership Styles in Public and Private Sector Universities: A Study in Pakistan" was retracted in 2025. Reason: plagiarism.

These findings highlight the importance of considering the organizational context and environment when examining leadership styles. The contrasting leadership styles observed in public and private sector universities suggest that leaders adapt their styles based on the specific demands and expectations of their respective sectors. The differences in attitudes towards leadership styles between the two sectors also have implications for job performance perceptions. Further exploration is warranted to understand how these differences in leadership styles may impact the motivation, engagement, and performance outcomes of followers in public and private sector universities. Additionally, investigating the factors that contribute to the variations in leadership styles and attitudes, such as organizational culture, institutional policies, and individual characteristics, can provide valuable insights for leadership development programs and strategies in both sectors.

Overall, these findings shed light on the distinctive leadership landscape within public and private sector universities about female leaders. Understanding these differences can help universities and educational institutions create supportive environments that foster effective leadership and enhance overall organizational performance. Thus, female leaders use both leadership styles according to the nature of the situation because, in the Pakistani context, subordinates are less motivated and lack knowledge and skills regarding innovation. So, in said environment, females have to use both leadership styles considering the situation. Thus, female leaders using transformational and transactional styles can establish a positive link with their subordinates and improve their performance by achieving the university's goals. These findings are in line with the findings of [49] which exposed a positive link between transformational leadership style and team performance similarly, the findings of [50]; and [47] were linked with the results of this investigation because their studies also discovered a link between both leadership styles and job performance.

[51] stated that the positive association between identity leadership and group-based pride is stronger when the leader political skill is advanced. Politically skilled leaders can access innumerable evidence and effectively convey influence on followers so that identity leadership has a robust effect on the pride of groups in the team. Therefore, leader political skill strengthens the indirect effect of group-based pride by which identity leadership improves team performance. So, leader political skill promotes the effectiveness of identity leadership in affecting team outcomes. Our results are reliable with these findings and endorse that managers should involve in more identity leadership behaviors to obtain better work results. Furthermore, identity leadership needs boundary conditions to produce more positive team performance. Politically skilled leaders can access to various information and deliver to their ideas to followers effectively, which strengthens the positive effect of identity leadership. Consequently, managers can increase their political skills to improve their inspiration on group members [9]. analysis showed that transformational and transactional leadership are closely related to employees' job performances which also supports the findings of this study.

The article "Comparative Analysis of Female Leadership Styles in Public and Private Sector Universities: A Study in Pakistan" was retracted in 2025. Reason: plagiarism.

## 7 Conclusion

In conclusion, this study highlights significant differences between female leaders in public and private sector universities in terms of their attitudes toward transformational leadership, transactional leadership, and job performance. Female leaders in public sector universities demonstrated a higher attitude towards practicing both transformational and transactional leadership styles, as well as job performance, compared to female leaders in private sector universities who exhibited a moderate attitude towards these factors. Interestingly, when comparing female leaders across different positions, no significant differences were found in their adoption of transformational leadership, transactional leadership, and job performance. This suggests that leadership styles and performance expectations may be consistent across various positions held by female leaders in both sectors.

Qualitative data further supported the understanding that female leaders possessed clear knowledge and understanding of both leadership styles and their role in achieving job performance. This underscores the importance of providing comprehensive training, workshops, and courses to empower and equip female leaders with the necessary skills and knowledge related to transformational and transactional leadership styles. In light of these findings, it is recommended that universities and educational institutions implement targeted interventions to enhance the leadership capabilities of female leaders. Such interventions can include training programs focused on developing transformational and transactional leadership skills, fostering a supportive organizational culture, and creating opportunities for networking and mentorship. By investing in the development of female leaders and their understanding of effective leadership styles, universities can harness the potential of their leaders to drive positive change, foster innovation, and improve overall job performance. Ultimately, this can contribute to the advancement of the education sector and facilitate the achievement of organizational goals in both public and private sector universities in Pakistan.

The article "Comparative Analysis of Female Leadership Styles in Public and Private Sector Universities: A Study in Pakistan" was retracted in 2025. Reason: plagiarism.

## Limitation and Future Direction

The study may have a limited sample size, which could affect the generalizability of the findings to a broader population of universities in Pakistan. Additionally, this study may not account for specific contextual factors that influence leadership styles, such as cultural, organizational, or regional differences. In future research we can extend the research to include a comparative analysis of female leadership styles in universities across different countries, considering cultural, social, and organizational factors. Moreover, we will investigate the impact of different leadership styles on organizational outcomes, such as employee satisfaction, performance, and organizational effectiveness. We can also explore the role of mentoring programs and support mechanisms in developing and nurturing female leaders in both public and private sector universities. Last but not least, we can consider the intersectionality of gender with other factors such as race, ethnicity, and socio-economic background to understand how these factors shape the experiences and leadership styles of female leaders in universities.

## Data Availability Statement

The original contributions presented in the study are included in the article/supplementary material; further inquiries can be directed to the corresponding author/s.

## Ethical Considerations

“Comparative Analysis of Females’ Leadership Styles of Public and Private Sector Universities in Pakistan This research study was carried out in the Punjab Province, Pakistan” Ethical consideration has been followed by the researcher in each step of the research. The Ethics Committee members of the School of Education Huanggang Normal University, Huanggang Hubei, China. Waived the need for ethics approval. The researcher enclosed the participant consent form with the questionnaire. All the participants of the study were informed about the purpose of the research and necessary permission taken before data collection the researcher assured the participant in his consent form that all information was collected, used only for academic purposes, and kept confidential. During data collection, the researcher considers all ethical issues related to females' aspects.

The article "Comparative Analysis of Female Leadership Styles in Public and Private Sector Universities: A Study in Pakistan" was retracted in 2025. Reason: plagiarism.

## Funding Statement

This research did not receive any specific grant from funding agencies in the public, commercial, or not-for-profit sectors.

## Additional Information

No additional information is available for this paper.

## CRediT authorship contribution statement

**Uzma Sarwar:** Formal analysis, Data curation, Conceptualization. **Rameez Tariq:** Resources, Project administration, Methodology. **Muhammad Aamir:** Validation, Supervision, Software. **Yurong Guan:** Writing – review & editing, Visualization.

## Declaration of Competing Interest

The authors declare that they have no known competing financial interests or personal relationships that could have appeared to influence the work reported in this paper.

## References

[1] Othmen J., Mohammed K.A., D'Silva J.L. (2012). Does a transformational and transactional leadership style predict organizational commitment among public university lecturers in Nigeria?. Asian Soc. Sci..

[2] Rehman S., Shareef A., Mahmood A., Ishaque A. (2014). Perceived leadership styles and organizational commitment. Interdiscipl. J. Contemp. Res. Bus..

[3] Abaslim U.D., Gberevbie D.E., Osibanjo O.A. (2018). 14th European Conference on Management, Leadership, and Governance.

[4] Dariush L., Choobdar G., Valadkhani P., Mehrali E. (2016). Leader facilitating organizational commitment of employees (Tehran). International Journal of Economics, Commerce and Management.

[5] Yasir M., Imran R., Irshad M.K., Mohamad N.A., Khan M.M. (2016). Leadership styles in relation to employees' trust and Organizational Change Capacity. Sage Open.

[6] Hoobler J.M., Masterson C.R., Nkomo S.M., Michel E.J. (2018). The business case for women leaders: meta-analysis, research critique, and path forward. J. Manag..

[7] Ward S. (2020). Leadership definition. The Balance Small Business; The Balance.

[8] Kabeyi J.B. (2018). Transformational vs. Transactional leadership with examples. Int. J. Bus. Manag..

[9] Thanh N.H., Quang N.V. (2022).

[10] Alnesr B., Ramzani S. (2019). The impact of transformational leadership on innovation through the mediating role of knowledge sharing in public and private universities of Syria. J. Bus. Manag..

[11] Demirtas O., Karaca M. (2020).

[12] Hasan E., Khajeh A., Abu M., Asaari H. (2018). Impact of leadership styles on organizational performance. J. Hum. Resour. Manag. Res..

[13] Kalsoom Z., Khan M.A., Zubair S.S. (2018). Impact of transactional leadership and transformational leadership on employee performance: a case of FMCG industry of Pakistan impact of transactional leadership and transformational leadership on employee performance: a case of FMCG industry of Pakistan. Ind. Eng. Lett..

The article "Comparative Analysis of Female Leadership Styles in Public and Private Sector Universities: A Study in Pakistan" was retracted in 2025. Reason: plagiarism.

[14] Othman F.S., Saad M.S.M., Robani A., Abdullah A.N. (2017). A conceptual framework of the impact of leadership styles on heterogeneous R& D team performance. International Symposium on Research in Innovation and Sustainability.

[15] Chaimongkonrojna T., Steane P. (2015). Effectiveness of full range leadership development among middle managers. J. Manag. Dev..

[16] Kim D., Choi C. (2014). Developing future leaders at Hyundai Motor Company through blended learning. Ind. Commerc. Train..

[17] Akram H. (2020). Education governance in Pakistan: a critical analysis. J. Soc. Sci. Adv..

[18] UNDP (2020).

[19] Khan I.U., Idris M., Amin R.U. (2021). Leadership style and performance in higher education: the role of organizational justice. Int. J. Leader. Educ..

[20] Northouse P.G. (2016).

[21] Grosso F.A. (2018).

[22] Naguni S., Sleegers P., Denessen E. (2016). Transformational and transactional leadership effects on teachers' job satisfaction, organizational commitment, and organizational citizenship behavior in primary schools: the Tanzanian case. Sch. Effect. Sch. Improv..

[23] Burns J.M. (1978).

[24] Bass B.M. (1985).

[25] Bass B.M., Avolio B.J., Chemmers M.M., Ayman R. (1993). Leadership Theory and Research: Perspectives and Directions.

[26] Bass B.M., Avolio B.J. (2004). Manual and Sampler Set.

[27] Kuhnert K.W., Bass B.M., Avolio B.J. (1994). Improving Organizational Effectiveness through Transformational Leadership.

[28] Bass B.M., Avolio B.J. (1990). The Implications of transactional and transformational leadership for Individual, team, and organizational development. Res. Organ. Change Dev..

[29] Boada M., Gutierrez J., Patiño T., Ríos M. (2023). Analysis of female participation in management positions: leadership styles in companies in the city of loja, Ecuador. Open J. Bus. Manag..

[30] Liao Xiaoyu, Lyu Bei, Fan Jiayu (2021). Gendered actual controlling shareholders and family business emotional attachment influences on business operational violations: a propensity score matching analysis. J. Psychol. Afr..

[31] Afshari L. (2022). Idealized influence and commitment: a granular approach in understanding leadership. Person. Rev..

[32] Avolio B.J., Bass B.M., Jung D.J. (1999). Re-examining the components of transformational and transactional leadership using the multifactor leadership questionnaire. J. Occup. Organ. Psychol..

[33] Bass B.M., Avolio B.J., Bass B.M., Avolio B.J. (1994). Improving Organizational Effectiveness through Transformational Leadership.

[34] Bass B.M., Riggio R.E. (2006).

[35] Levine M.F. (2000).

The article "Comparative Analysis of Female Leadership Styles in Public and Private Sector Universities: A Study in Pakistan" was retracted in 2025. Reason: plagiarism.

[36] Su W., Lyu B., Chen H., Zhang Y. (2020). How does servant leadership influence employees' service innovative behavior? The roles of intrinsic motivation and identification with the leader. Baltic J. Manag..

[37] Chron C. (2020). The four elements of transformational leadership. Leadership.

[38] Bass B.M. (1998).

[39] Gill R. (2006).

[40] Bass B.M., Steidlmeier P. (1999). Ethics, character, and authentic transformational leadership Behavior. Leader. Q..

[41] House R.J., House R.J., Hanges P.J., Javidan M., Dorfman P.W., Gupta V., Associates (2014). Culture, Leadership, and Organizations: the GLOBE Study of 62 Societies.

[42] Bass B.M. (1999). Two decades of research and development in transformational leadership. Eur. J. Work. Organ. Psychol..

[43] Motowidlo S.J., Kell H.J. (2012). Chapter 5 job performance. Handbook of Psychology.

[44] Deslie N. (2015). The impact of leadership style on employee performance. J. Manag. Dev..

[45] Pawirosumarto S., Sarjana P., Muchtar M. (2017). Factors affecting employee performance of PT.Kiyokuni Indonesia. International Journal of Law and Management.

[46] Stump M.N. (2013).

[47] Wood T.B. (2019). An examination of the suitability of transactional, transformational and situational leadership theories in evaluating the role of gender in determining the leadership style: a comparison and contrast of three leadership theories. Am. J. Manage. Stud..

[48] Bass B., Avolio B. (1995). MLQ multifactor leadership questionnaire.

[49] Jaroliya D.D., Gyanchandani R. (2021). "Transformational leadership style: a boost or hindrance to team performance in IT sector". Vilakshan-XIMB. J. Manag..

[50] Buil I., Martinez E., Matute J. (2019). Transformational leadership and employee performance: the role of identification, engagement and proactive personality. Int. J. Hospit. Manag..

[51] Hou L., Song L.J., Zheng G., Lyu B. (2021). Linking identity leadership and team performance: the role of group-based pride and leader political skill. Front. Psychol..

[52] Cascio W.F. (1995). Whither industrial and organizational psychology in a changing world of work. Am. Psychol..

[53] Dastoor B., Suwannachin K., Golding A. (2013).

[54] Downton J.V. (1973).

[55] Hargis M.B., Watt J.D., Piotrowski C. (2011). Developing leaders: examining the role of transactional and transformational leadership across contexts business. Organ. Dev. J..

[56] Hater J.J., Bass B.M. (1988). Superiors' evaluation and subordinates' perception of transformational and transactional leadership. J. Appl. Psychol..

[57] House R.J., Hunt J.G., Larson L.L. (1976). Leadership: the Cutting Edge. *A Symposium Held at Southern Illinois University*.

[58] House R., Woychke J., Fodo E., Conger J., Kanungo R. (1988). Emerging Leadership Vistas.

The article "Comparative Analysis of Female Leadership Styles in Public and Private Sector Universities: A Study in Pakistan" was retracted in 2025. Reason: plagiarism.

[59] Kirkman B., Chen G., Farh J.L., Chen Z.X., Lowe K. (2009). Individual power distance orientation and follower reactions to transformational leaders: a cross-level, cross-cultural examination. Acad. Manag. J..

[60] Nanjundeswaraswamy T.S., Swamy D.R. (2014). Leadership styles. A review paper. Advances in Management.

[61] Pakistan Economic Survey (2019).

[62] Pradhan R., Jena L. (2016). Employee performance at workplace: conceptual model and empirical validation. Business Perspectives and Research.

[63] Torlak N.G., Kuzey C. (2019). Leadership, job satisfaction and performance links in private education institutes of Pakistan. Int. J. Prod. Perform. Manag..

[64] Wen T.B., Ho T.C.F., Kelana B.W.Y., Othman R., Syed O.R. (2019). Leadership styles in influencing employees' job performances. Int. J. Acad. Res. Bus. Soc. Sci..

